# Study on the Prognosis Effect of Traditional Chinese Medicine Treatment in DR Patients Based on the Perspective of Network Pharmacology

**DOI:** 10.1155/2022/3528732

**Published:** 2022-07-19

**Authors:** Xiaoyuan Man, Zijin Sai

**Affiliations:** ^1^Shandong University of Traditional Chinese Medicine, Jinan 250355, China; ^2^Weihai Hospital of Traditional Chinese Medicine, Shandong University of Traditional Chinese Medicine, Jinan 250355, China

## Abstract

Diabetes damages the eye in many ways, but the most common eye complication is retinopathy. Of the 246 million people with diabetes worldwide, about 30% will be at risk of developing diabetic retinopathy. In addition to impairing vision, the presence of diabetic retinopathy also means an increased risk of life-threatening systemic vascular complications. To prevent the occurrence and development of diabetic retinopathy, the research and development of new drugs for diabetic retinopathy is the primary task. Because of its characteristics of holistic view and dialectical view, traditional Chinese medicine has a good effect in the treatment of complex diseases. However, due to the characteristics of complex components, numerous targets, and synergistic effects that are important, and its compound prescriptions, the modernization of traditional Chinese medicine has been hindered. The rise of network pharmacology in recent years provides a good opportunity for the development of traditional Chinese medicine. Network pharmacology aims to explore the relationship between drugs and diseases from a holistic perspective, discover drug targets, and guide the development of new drugs. In terms of methodology, network pharmacology has the characteristics of integrity and systematicness, which just coincides with the principle of consultation in traditional Chinese medicine. In this paper, from the perspective of the application of traditional Chinese medicine, TCMSP software was used to retrieve the active ingredients in traditional Chinese medicine, and the corresponding targets of the active ingredients were obtained. We then performed GO annotation analysis and KEGG pathway analysis on the targets using DAVID software. We further used Cytoscape software to build an active ingredient-target-pathway network model. Through network pharmacology research, it has been shown that Fufang Xueshuantong may treat diabetic retinopathy through multiple pathways such as intravascular growth factor signaling pathway, mitogen-activated protein kinase signaling pathway, and Toll sample receptor signaling pathway, reflecting the multicomponent traditional Chinese medicine compound and multitarget and multichannel characteristics. The research in this paper provides a theoretical basis for the pharmacological mechanism of traditional Chinese medicine in the treatment of diabetic retinopathy.

## 1. Introduction

Diabetes mellitus is a common endocrine disease dominated by glucose metabolism disorders, and the prevalence of diabetes and the number of diabetic patients are increasing rapidly [1–4]. The International Diabetes Federation estimates that, by 2040, 1 in 10 adults (20–79 years old) will be diagnosed with diabetes. In 2045, there will be 629 million people with diabetes worldwide, and the death rate from diabetes will be greater than the death rate from AIDS, tuberculosis, and malaria combined. By 2045, about 5 million people will die of diabetes each year, or about 1 person with diabetes dies every 6 seconds. According to statistical forecasts, the total global diabetes health care expenditure is expected to grow to 802 billion US dollars by 2040. According to the research data of the Chinese National Health and Family Planning Commission's “Diabetes Prevention and Control in China,” as of 2019, the number of people with diabetes in my country is about 116 million, and the overall diabetes prevalence rate is 9.7%, ranking first in the world. As shown in Figure 1, the study predicts that the number of people with diabetes in my country will reach 151 million in 2024, which is equivalent to 1 in 14 people suffering from diabetes.

As the duration of diabetes increases, the risk of various complications caused by diabetes also increases, and the most serious complication is Diabetic Retinopathy (DR). Diabetic retinopathy is one of the three major eye diseases that cause blindness in humans, and it is caused by diabetes. When diabetic patients have poor blood sugar control, the blood will flow through various blood vessels and organs in the body with high concentrations of blood sugar. When excess sugar flows into the fundus and retina, it is very likely that polysaccharide particles will form to block the capillaries in the fundus, preventing normal blood flow. Long-term blockage will cause local hypoxia and rapid reduction of hemoglobin in the retinal tissue, and further risk of blood vessel rupture, which may eventually lead to visual impairment or even blindness in patients [5–8]. According to statistics, about one-third of diabetic patients in China suffer from diabetic retinopathy. If the patient cannot be diagnosed and treated in the early stage of the disease, it is likely to cause visual impairment or even blindness. The damage to vision caused by diabetic retinopathy is irreversible. Early detection and timely medical treatment are the best treatment methods. Therefore, early screening and diagnosis of diabetes is of great significance [9]. The occurrence and development of diabetic retinopathy affect people's life to a great extent and also affect people's quality of life. The course of diabetes, blood glucose level, blood pressure, blood lipids, and other clinical factors have certain influence on the occurrence and development of diabetic retinopathy. There are great individual differences in the course and severity of diabetic retinopathy. Some patients with long-term diabetes do not develop diabetic retinopathy despite poor glycemic control, while others develop diabetic retinopathy rapidly. The above differences may be due to genetic polymorphisms. In recent years, there has been an increase in the understanding of the safety and biodistribution of gene delivery vectors. Studies have shown that stem cell and gene therapy can reverse degenerative retinopathy. Drugs involve regeneration of atrophic or damaged retinal tissue, neurotrophic factors, immunomodulation, and new therapies that replace mutated genes. With the advancement of science and technology, the number of genes that can be selected for intervention has gradually increased. The current gene therapy research for diabetic retinopathy is to use related gene drugs against pigment epithelium-derived factor, angiostatin, endostatin, and vascular endothelial growth factor, inhibit endothelial cell proliferation, and form new blood vessels, with these to achieve the clinical purpose of prevention and treatment of diabetic retinopathy. At present, the pathogenesis of diabetic retinopathy and related genes still needs to be further explored.

Diabetes has a thousand years of history in Chinese medicine. Diabetes is the closest to diabetes in Chinese medicine. In modern medicine, the two are often equated. DR belongs to diabetes mellitus cancer. Most physicians call DR the diabetes mellitus disease, which belongs to the categories of bird's eye, cataract, and violent blindness. Liver and kidney deficiency and heart and spleen deficiency lead to eye orifice dystrophy. After many clinical practices, it has been proved that traditional Chinese medicine has a significant effect in the prevention and treatment of diabetic retinopathy. However, it also faces the relatively slow theoretical research on traditional Chinese medicine compounds due to the complex components and unclear mechanism of action. Moreover, it is difficult to achieve the preset purpose by using traditional pharmacological experimental methods. With the gradual improvement of systems biology and the vigorous development of network pharmacology combined with computer technology, multidisciplinary research methods have emerged. These methods have been gradually applied in the field of traditional Chinese medicine. The emergence of these emerging scientific technologies has provided new methods and strategies for exploring the theory, clinical research, and drug development of diabetic retinopathy. The research mode of network pharmacology has also changed from single drug and single target to disease-gene-target-drug. The overall analysis of the biological system network, the prediction of the pharmacological mechanism of the drug, and the evaluation of the clinical effect of the drug are helpful for the related research of traditional Chinese medicine compounds and the development of new multitarget traditional Chinese medicine drugs.

Network pharmacology has the characteristics of integrity and system, which is in harmony with the holistic view of traditional Chinese medicine and the principle of dialectical treatment. This article briefly reviewed the opportunities and challenges of the modernization of traditional Chinese medicine and the generalization of the formation of network pharmacology. On this basis, the network pharmacology method was used to analyze the drug-target-disease relationship of traditional Chinese medicine in the treatment of diabetic retinopathy, and to corroborate the biological mechanism of highly expressed genes. The research in this paper can provide a basis for further clinical research on diabetic retinopathy.

## 2. Related Work

### 2.1. Research Status of Diabetic Retinopathy

The retina is a transparent and soft membrane, which is located behind the inner wall of the eyeball. It is rich in blood vessels and is the only blood vessel that the human body can see. In clinical practice, doctors use the retinal images of the fundus to judge the changes in the blood vessels of the patient's body. The retina contains tissues such as the macula, optic disc, and blood vessels. The optic disc, also known as the optic disc, is the initial end of the optic nerve and is in the shape of a reddish disc. The macula is located on the temporal side of the optic disc and is darker than the surrounding retinal area, with a depression in the center of the macula called the fovea. As shown in Figure 2, the red and slender lines in the retina are the blood vessels of the fundus. The retina of the healthy fundus is light orange, the border of the optic disc is clearly visible, and the blood vessels are clearly filled [10]. When diabetic patients develop retinopathy, some pathological changes will occur in the retinal area, and different disease degrees correspond to different disease characteristics. Usually, the main features of diabetic retinopathy are microaneurysms, bleeding spots, hard exudates, soft exudates, hyperplastic blood vessels, and so on. Microaneurysms, which usually appear early in the disease process, are dark red dots on the retina due to thinning of the blood vessel walls due to lack of oxygen in the capillaries of the eye. Bleeding spots generally appear near the blood vessels, which are formed by blood oozing due to vascular blockage, and appear as dark spots. The formation of soft and hard exudates indicates that the lesion has reached a relatively severe level. When the blood supply is poor for a long time, the terminal capillaries will be necrotic, and this part of the necrotic blood vessels will show large-scale bright spots or flocs on the retina. When the eyeball is in a state of hypoxia for a long time, the eyeball will proliferate new blood vessels to obtain oxygen and blood [11–13].  Figure 3 shows the retinal fundus image of the lesion, which contains the main lesion features. Diabetic retinopathy is one of the most common and serious chronic microvascular complications of diabetes. DR is usually divided into nonproliferative and growth phases. Harm of DR: there are generally no ocular adaptive symptoms in the early stage of the disease. With the aggravation of the disease, the regulation function of the blood vessels itself becomes abnormal, and the vision is severely reduced, which may eventually lead to blindness. DR is one of the leading causes of blindness worldwide. All people with diabetes are at risk for DR. The longer a patient has diabetes, the higher the chance of developing DR is. The pathogenesis of DR is complex, and the common starting point is hyperglycemia. It is generally believed that DR is caused by damage to the blood-retinal microvascular system. The increased production of free radicals in retinal tissue cells is due to the long-term exposure of cells to a high-glucose environment, and vascular endothelial cells will generate a large amount of reactive oxygen species (ROS) under the stimulation of a high-glucose environment.

Endothelial cells, pericytes, and basement membrane together make up retinal capillaries. Endothelial cells participate in the immune activity of the body, which can affect vasoconstriction and vasodilation and regulate local blood flow and vascular permeability in retinal capillaries. Endothelial cells connect with pericytes to form the blood-retinal barrier and maintain the stability of retinal capillaries. Pericytes can also regulate the permeability of local blood flow in retinal capillaries and can also provide support for endothelial cells and inhibit endothelial cell proliferation. It has been reported that the activity of antioxidant enzymes in retinal tissue decreases during hyperglycemia, resulting in the accumulation of a large amount of ROS in vascular endothelial cells and pericytes, resulting in oxidative stress. Under normal biological conditions, ROS remain in balance, but their overproduction can lead to a biological process called oxidative stress, which is considered to be the main pathogenesis of DR. ROS can damage intracellular biomacromolecules, cause increased oxidative stress, and ultimately lead to mitochondrial dysfunction and retinal cell apoptosis.

### 2.2. Understanding of Traditional Chinese Medicine on Diabetic Retinopathy

The pathogenesis of DR is complex. Although there is no cure for traditional Chinese medicine, traditional Chinese medicine has great advantages in conservative treatment of DR. Traditional Chinese medicine can improve vision and delay the development of DR, which reflects the broad prospects and unique advantages of traditional Chinese medicine in the treatment of DR. In terms of treatment, traditional Chinese medicine pays more attention to the functions of regulating qi and activating blood, nourishing the liver and kidney. Studies have confirmed that, in the process of DR development, blood stasis has always been an important pathogenesis of DR, so the method of promoting blood circulation and removing blood stasis is one of the effective means of treating DR. There are many reasons for blood stasis: yin deficiency, qi and blood stasis, phlegm-dampness caused by blood stasis, blood heat caused by blood stasis, etc. Traditional Chinese medicine summarizes DR as endogenous dryness and heat, yin deficiency constitution; or inappropriate diet, causing damage to the spleen and stomach; or excessive fatigue and insufficient yin. Deficiency of both qi and yin and deficiency of liver and kidney can cause vision loss; dry eyes and long-term high sugar conditions can lead to microvascular disease. At the same time, yin deficiency and dryness heat will make the blood flow not smooth, and blood stasis will endogenously lead to blockage of the eyes and collaterals, which will aggravate DR [14]. Since ancient times, traditional Chinese medicine has achieved good results in preventing and treating the complications of diabetes. Traditional Chinese medicine has low toxicity, small side effects, mild effect, and long-lasting efficacy. Many traditional Chinese medicines can effectively prevent and alleviate diabetes and its complications while lowering blood sugar [15]. At present, it is found that Chinese herbal medicines are needed to effectively prevent and delay the occurrence of DR, and astragalus is the first choice for the treatment of DR. *Astragalus* is a qi-tonifying medicine with a lukewarm nature. DR often has the phenomenon of yin deficiency and qi deficiency. *Astragalus* belongs to the spleen and lung and has the effect of tonifying qi. Studies have confirmed that astragaloside IV in *Astragalus* has anti-inflammatory and antioxidant effects and has a preventive effect on DR and balances oxidative stress responses. *Astragalus* polysaccharides can be anti-inflammatory and antioxidant, reduce VEGF expression, and reduce the adhesion of leukocytes to the retina, thereby preventing and treating DR. *Panax notoginseng* can remove blood stasis and stop bleeding, warm in nature, and return to the liver and stomach. It has the effect of stopping bleeding without leaving stasis. *Panax notoginseng* can reduce retinal vascular permeability, decrease blood viscosity, protect capillary structure, and delay the development of DR. The study found that the traditional Chinese medicine Ginkgo biloba, Pueraria, Angelica, and its extracts significantly improved many indicators of DR patients.

At present, many Chinese patent medicines are developed by some Chinese medicine compounds, which improves the patient's compliance and provides convenience for patients to take medication under certain conditions. There are many compound Chinese patent medicines used for the treatment of DR in clinic, including tablets, capsules, and granules. There are also many corresponding clinical trials.

### 2.3. Combination and Application of Network Pharmacology and Modernization of Traditional Chinese Medicine

The medical treatment is guided by the holistic view and dialectical treatment, and the traditional Chinese medicine compound formula with the compatibility principle of “monarch, minister, assistant, and envoy” is the main form of clinical disease prevention and treatment. Based on the characteristics of integrity and dynamics, Chinese network pharmacology advocates the principle of multitarget and multichannel drug delivery. Therefore, in the process of TCM modernization, some TCM researchers draw on the research ideas of network pharmacology to explore the essential attributes of TCM “prescriptions for symptoms.” These essential attributes reveal the multichannel, multitarget, and multicomponent comprehensive effects of traditional Chinese medicine and its compounds, and good staged results have been achieved. The basic characteristics of traditional Chinese medicine lie in the holistic view and dialectical treatment, and it is characterized by the combination of diseases and the corresponding prescriptions and syndromes, that is, the diagnosis and treatment mode of “disease prescription.” Symptoms are the core content of the characteristic diagnosis and treatment system of traditional Chinese medicine, which is the holistic view, dialectical treatment, and compound intervention. The difference between dialectical treatment and “symptom” treatment is that the former treats the “symptom” that reflects the overall change, while the latter treats the symptoms point-to-point. On the cognitive level, the latter is shallower and belongs to perceptual cognition; the former is deeper, with a leap from perceptual cognition to rational cognition, which is the stage of cognition that goes deep into the internal laws of things. Elucidating the biological basis of symptoms is one of the keys to the modernization of traditional Chinese medicine. Decades of modern research on symptoms have shown that symptoms are complex systems composed of many factors, which are difficult to express with a single physiological and biochemical index. Therefore, with the increase of research depth and complexity, it is necessary to develop a suitable way to discover TCM symptom characteristics from complex systems. Network pharmacology integrates the information of “disease-phenotype-gene-drug” to understand the relationship between disease phenotype and life macromolecules from a systematic perspective. Its idea of “disease phenotype-biomolecule” network construction serves to guide the research on the biological basis of TCM symptoms. Many researchers have carried out research on the biological basis of syndromes from the perspective of biomolecular networks, formed a research framework suitable for interpreting the connotation of the system of disease-syndrome prescriptions, and further proposed the concept of biomolecular network markers for syndromes. Through network function analysis, the researchers found that the biomolecular network of cold syndrome is dominated by the functional modules of hormones, the biomolecular network of heat syndrome is dominated by the functional modules of cytokines, and the functional modules of neurotransmitters are distributed in the two networks. The researchers also analyzed the possibility of applying syndrome molecular network markers to research fields such as syndrome objectification and individualized diagnosis and treatment, clinical effect evaluation of traditional Chinese medicine, prescriptions, and medicinal properties of traditional Chinese medicine.

Pharmacodynamic substances in traditional Chinese medicine refer to the chemical composition system that exerts pharmacological effects in traditional Chinese medicines and compound prescriptions. The pharmacodynamic material basis of traditional Chinese medicine cannot be attributed to a specific effective chemical component, and its mechanism of action does not act on a specific target but is the result of the overall regulation of multiple components through multiple targets and multiple links. In network pharmacology, a drug-drug network can be constructed based on the similarities between drugs and drugs in terms of structure and efficacy, and the efficacy of drugs and the chemical composition of efficacy can be predicted. This method of network pharmacology can also be applied to the prediction of the efficacy of effective and effective components of traditional Chinese medicine and the analysis of the chemical components of the effective substances. Many studies [16, 17] predicted, understood, and clarified the pharmacodynamic substances of traditional Chinese medicines from the perspective of the network, which provided a good reference and inspiration for the in-depth research on the pharmacodynamic substances of traditional Chinese medicines. The research on the modernization of traditional Chinese medicine is also inseparable from the revealing of the mechanism and law of action of traditional Chinese medicine. The curative effect of traditional Chinese medicine compound is the result of the interaction between the various pharmacodynamic substances and the macromolecules of the body. The multicomponents of traditional Chinese medicine and its compound determine the multitarget and multilink of its action, and the effects of different components on different links finally show changes that are beneficial to the body. Network pharmacology is a theory that studies multitargets to intervene disease networks and achieve ideal drug efficacy. It can be seen that the drug delivery ideas of network pharmacology and the compound drug delivery of traditional Chinese medicine have the same purpose. The technical method of network pharmacology can be well applied to the study of the mechanism of action of traditional Chinese medicine. Xu et al. [18] used the means of network pharmacology, using molecular docking and complex network analysis techniques to study the interaction between the chemical components and targets in traditional Chinese medicine for the treatment of chronic kidney disease. The results showed that the chemical composition-target interaction network contained in traditional Chinese medicine for the treatment of chronic kidney disease was quite different from that of western medicine. This shows that the mechanism of action of traditional Chinese medicine is not exactly the same as that of western medicine. Their research also found that the chemical component-target interaction network contained in tonic Chinese medicines is also quite different from the chemical component-target interaction network contained in other types of Chinese medicines. This explains the ancient theory of traditional Chinese medicine from the perspective of complex network research. At the same time, they used molecular docking method to study the interaction of these 1729 compounds with 26 recognized targets related to cardiovascular diseases and their distribution in the target space, elucidating the possible mechanism of Qishen Yiqi Dropping Pills in the treatment of vascular diseases, active molecules.

## 3. Materials and Methods

Firstly, the chemical constituents of *Panax notoginseng*, *Astragalus*, *Salvia miltiorrhiza*, and Scrophulariaceae were retrieved from Traditional Chinese Medicine Systems Pharmacology Database and Analysis Platform (TCMSP) database to collect chemical constituents-target information. The DR-related targets were then retrieved from the database of five disease-related targets, OMIM, TTD, pharmGkb, DiGSeE, and GAD. DiGSe is an online text mining tool that can mine disease-related genes. Using the Uniprot database, input the target name obtained from TCMSP and 5 databases to obtain the corresponding gene name and correct the protein name. We preferentially select gene names that are included in Swiss-prot and have a high degree of matching. The intersection of Fufang Xueshuantong and DR-corrected genes were obtained. Next, Gene ontology (GO) annotation analysis and Kyoto encyclopedia of genes and genomes (KEGG) were performed on the obtained intersection genes using the DAVID database. Intersection genes can be directly mapped onto pathways. According to the target prediction results of the above chemical components of Fufang Xueshuantong, Cytoscape software was used to construct a chemical component-intersection target-pathway network model. In the network, nodes represent chemical components, intersecting genes and pathways. If a target is a potential target of a compound, it is connected by an edge. When the target is involved in a certain pathway, the target and the action pathway are also connected by an edge. The multicomponent, multitarget, and multipathway characteristics of Fufang Xueshuantong in the treatment of DR were revealed by constructing a network. We used UniProt search to select the PDB ID of the appropriate target. The 3D structure files of the docking protein and control ligands were downloaded using RSCB PBD, where the control ligands were automatically matched by the RSCB PBD system. Then, use PubChem to download the 3D structure file of the compound, and finally use the SystemsDock online molecular docking tool for online molecular docking.

## 4. Results

### 4.1. Collection of Chemical Components and Target Genes

We retrieved and found that there are 119 chemical constituents of *Panax notoginseng*, 202 kinds of *Salvia miltiorrhiza*, 87 kinds of *Astragalus* root, and 47 kinds of Scrophulariaceae. A total of 427 chemical components were deleted, including compounds such as flavonoids, terpenoids, glycosides, carbohydrates, fatty acids, and amino acids, such as luteolin, apigenin, dehydrotanshinone II, salvianolic acid b, ursolic acid, and L-lysin (numbered as 6 , 8, 2651, 7074, 511, and 55). Some researchers measured the main chemical components in Fufang Xueshuantong capsule by UPLC-MS/MS method and found that the contents of tanshinone II-A, salvianolic acid B, and ursolic acid were 1.135, 2.343, and 0.560 (mg/g), respectively. The chemical components of Fufang Xueshuantong correspond to 376 genes, such as VEGF, mitogen-activated protein kinase 8, MAPK8, and IL-1*β*.

### 4.2. DR-Related Target Pathway Information

A total of 247 DR-related genes were obtained from 5 databases, including vascular endothelial growth factor A, MAPK1, and MAPK8. Through DAVID analysis, the Toll-like receptor signaling pathway, MAPK receptor signaling pathway, VEGF signaling pathway, and other pathway information were obtained, as shown in Table 1.

### 4.3. Biomolecular Functional Annotation of Intersecting Genes

The intersection of Fufang Xueshuantong target genes and DR-related genes showed that there were 37 identical genes, including VEGF, MMP, IL-1*β*, PTGS2, and MAPK8. We annotated the biomolecular functions of the 37 intersecting genes through the DAVID system and performed GO annotation analysis and KEGG pathway analysis on the acquired targets. The GO annotation analysis is divided into three parts, namely, molecular function, cellular component, and biological process. Among the molecular functions of the intersecting genes, the protein binding and heparin binding functions are the most involved. Related genes include JUN, SRC, and VEGFA. Intersection genes were most distributed in the extracellular space, cytosol, and cell surface. Genes such as superoxide dismutase, IL-6, and IL-1*β* are involved. Intersection genes and inflammatory response, positive regulation of RNA polymerase II promoter transcription, positive regulation of endothelial cell proliferation, and other biological processes are the most numerous. Genes such as NOS1, IL-1*β*, and VEGFA are involved.

### 4.4. Construction of Chemical Composition-Intersection Gene-Pathway Network

By KEGG analysis, a total of 18 pathways were obtained, including 24 intersection genes. Pathways were screened by the criterion of *P* < 0.05, and finally, 14 pathways and 22 genes were obtained. We used Cytoscape software to construct chemical component-gene-pathway network model. In this model, there are a total of 169 nodes and 458 edges. There are many effective chemical components acting on MAPK8, IL-6, IL-1*β*, and COX-2. These targets involve more pathways including TLR signaling pathway, MAPK signaling pathway, and VEGF signaling pathway. The chemical components acting on the above targets and pathways include luteolin, apigenin, ursolic acid, and K-lysine. The action targets of the main active components of Fufang Xueshuantong are distributed in different signaling pathways, which coordinate with each other and play a role together.

It has been reported in the literature that the mechanism of compound Xueshuantong in the treatment of DR mainly includes dilation of blood vessels, improvement of antihypoxia ability, inhibition of oxidative stress, and reduction of apoptosis. These findings are consistent with the network prediction results in this paper. This study can reveal the drug mechanism of Fufang Xueshuantong in the treatment of DR from multiple perspectives.

### 4.5. Construction of Chemical Composition-Intersection Gene-Pathway Network

Two targets of COX-2 and VEGFR2 were selected, and 5 compounds of luteolin, quercetin, kaempferol, and ursolic acid (No. 6, 8, 98, 422, and 511) and control ligands of 4 targets were selected for Molecular docking, as shown in Table 2. The results of molecular docking were consistent with the results predicted by network pharmacology in this paper. The docking scores of the five compounds numbered 6, 8, 98, 422, and 511 were significantly higher than those of the control ligand. The results indicated that the five compounds had good effects on COX-2 and VEGFR2.

## 5. Discussion

Fufang Xueshuantong in the treatment of DR has been clinically proven. However, the pharmacological mechanism of Fufang Xueshuantong in the treatment of DR is still unclear. In 2008, Hopkins clearly proposed the concept of network pharmacology. This paper uses the research ideas of network pharmacology to explore the potential targets and mechanisms of Fufang Xueshuantong in the treatment of DR and predict the possible targets and pathways of Fufang Xueshuantong in the treatment of DR.

Inflammation is the initial reaction of retinal blood vessels stimulated by high glucose, manifested as leukocyte aggregation and a large increase in the secretion of inflammatory factors. Neovascularization is the hallmark pathological feature of DR. In this paper, the analysis of DR-related genes found that VEGF signaling pathway, TLR signaling pathway, and MAPK signaling pathway play a central role in the process of inflammation and vascular proliferation. COX-2 is an important inducible enzyme in the inflammatory process. The promotion of angiogenesis by COX-2 may be related to its induction of tissue production of VEGF. VEFG specifically acts directly on endothelial cell surface receptors to promote angiogenesis. VEGFA is an important member of the VEGF family, which can promote neovascularization and increase vascular permeability.

VEGF signaling pathway, TLR pathway, and MAPK pathway coordinate with each other and influence each other. For example, both COX-2 and TLRs can induce tissue production of VEGFA, which binds to its receptor KDR and activates MAPK1/8 or c-Jun N-terminal kinase, thereby affecting the MAPK signaling pathway. MAPK is a regulator of FGF2-induced angiogenesis. FGF2 has chemotactic and mitotic effects on endothelial cells, promotes angiogenesis, and leads to angiogenesis. Studies have shown that both exogenous and endogenous FGFs can induce VEGF production and affect angiogenesis.

In this study, combined with the data analysis of TCMSP and DAVID, it was found that a total of 92 compounds, including luteolin, ursolic acid, quercetin, kaempferol, and apigenin, may have 21 targets for the above-mentioned 3 pathways. The data analysis in this paper found that, among the chemical components of Fufang Xueshuantong, one chemical component can correspond to multiple targets and participate in multiple signaling pathways. For example, the corresponding targets of ursolic acid in Scrophulariaceae are IL-1*β*, MAPK8, JUN, and MMP2, which regulate VEGF signaling pathway, TLR signaling pathway, and local adhesion. Moreover, in the pathogenesis of DR, multiple chemical components of Fufang Xueshuantong can also correspond to a common target, such as luteolin, apigenin, and ursolic acid, which act together on VEGFA.

In conclusion, this subject analyzed the components and targets of Fufang Xueshuantong and collected DR-related genes. We used network pharmacology to obtain the relevant pathways of the two intersection genes and predicted that Fufang Xueshuantong acts on multiple signaling pathways such as VEGF, TLR, and MAPK through multiple chemical components such as ursolic acid, quercetin, and kaempferol. This study shows that Fufang Xueshuantong is an important compound, and its chemical components may directly act on the key pathway targets of DR and treat DR by inhibiting inflammation and vascular proliferation. This study provides a typical basis for further revealing the typical pharmacological mechanism of traditional Chinese medicine, represented by compound Fufang Xueshuantong, in the treatment of DR.

## Figures and Tables

**Figure 1:** Number and forecast of diabetes patients in China from 2018 to 2024.

**Figure 2:** Fundus image of healthy retina.

**Figure 3:** Diseased retinal fundus images.

**Table 1:** The part of pathways and genes of diabetic retinopathy (DR).

Pathway	Count	Gene
*Salmonella* infection	6	MAPK1, IL6, JUN, IL1B, MAPK8, NOS2
VEGF signaling pathway	5	MAPK1, PTGS2, VEGFA, SRC, KDR
Focal adhesion	7	MAPK1, JUN, VEGFA, MET, MAPK8, SRC, KDR
Influenza A	6	MAPK1, IL6, JUN, IL-1*β*, MAPK8, PLG
GnRH signaling pathway	5	MAPK1, JUN, MAPK8, MMP2, SRC
Toll-like receptor signaling pathway	5	MAPK1, IL6, JUN, IL-1*β*, MAPK8
NOD-like receptor signaling pathway	4	MAPK1, IL6, IL-1*β*, MAPK8
MAPK signaling pathway	6	MAPK1, JUN, TP53, IL-1*β*, MAPK8, FGF2
ErbB signaling pathway	4	MAPK1, JUN, MAPK8, SRC
Herpes simplex infection	5	IL6, JUN, TP53, IL-1*β*, MAPK8
Cytokine-cytokine receptor interaction	5	IL6, VEGFA, MET, IL-1*β*, KDR
Arginine and proline metabolism	3	NOS1, ALDH2, NOS2
Regulation of actin cytoskeleton	5	MAPK1, INS, ITGB2, FGF2, SRC
Cell adhesion molecules (CAMs)	4	SELP, ITGB2, SELE
FoxO signaling pathway	4	MAPK1, IL6, INS, MAPK8
Glycerolipid metabolism	3	LPL, AKR1B 1, ALDH2
Adherens junction	3	MAPK1, MET, SRC
Progesterone-mediated oocyte maturation	3	MAPK1, INS, MAPK8

**Table 2:** The result of molecular docking.

Ligand	Cox-2	VEGFR2
The control ligand of cox-2 (tolfenamic acid)	1.454	—
The control ligand of VEGFR2 (C_14_H_23_N_5_O)	—	3.227
Luteolin (6)	6.725	6.628
Apigenin (8)	6.795	—
Quercetin (98)	6.597	6.354
Kaempferol (422)	6.679	6.374
Ursolic acid (511)	—	7.428

## Data Availability

The data underlying the results presented in the study are available within the article.
